The article "ECANP: A Topic Influence Evaluation Model for Hot Topics" was published in 2022. Journal: Comput Intell Neurosci.

# ECANP: A Topic Influence Evaluation Model for Hot Topics

**DOI:** 10.1155/2022/5943634

**Published:** 2022-06-30

**Authors:** Yiru Chang, Zhiyuan Zhang, Guixun Luo

**Affiliations:** ^1^School of Electronic and Information Engineering, Key Laboratory of Communication and Information Systems, Beijing Municipal Commission of Education, Beijing Jiaotong University, Beijing 100044, China; ^2^School of Computer and Information Technology, Beijing Jiaotong University, Beijing 100044, China

## Abstract

Social network is an important product of industrial society. In recent years, the research related to hot topics has focused on topic detection, topic trend prediction, and topic tracking. However, the important role of topic influence evaluation in hot topic research has not received enough attention, which leads the problem of inaccurate influence calculation. In order to solve the above problems, this paper proposes a novel model to evaluate the real-time relative influence of topics in social network. The proposed model can quantify the influence of topics, and some influential factors which determine topic hotness will be analyzed and identified. In this model, five impact indicators are defined, namely user engagement, topic coverage, topic activity, topic persistence, and topic novelty to consider the topic characteristics more finely. Moreover, the proposed model not only consider traditional simple factors of like, forward and comments, but also pay attention to the relative influence and time attenuation characteristics of the topics. Further, the experimental results show that our method could quickly aggregate the influence factors of hot topics and accurately provide the influence indicator of topics.

## 1. Introduction 

In the society of smart industry, the Internet has increasingly become a way of information dissemination that cannot be ignored. On the one hand, as the most timely and widest media for information access, the Internet has become the main channel for the central government, relevant government departments, and authoritative platforms to release news and access information [1]. On the other hand, due to its good interaction, various forms of expression, and outstanding appeal, it has not only attracted major websites and organizations to use it as a publicity channel, but also gained more and more users. By December 2021, the number of Internet users in China had reached 1.032 billion, and the Internet penetration rate had reached 73.0% [2], an increase of 1.4 percentage points over half a year ago. It can be seen that the Internet plays an extremely essential role in information dissemination and daily life.

The emergence of social media, especially the application of mobile communication technology, enables people to break the restrictions of time and space simultaneously, and garner, share, and exchange information from the Internet whenever and wherever possible, which led to an increasing number of Internet users and the rapid expansion of information on various platforms. In particular, Sina Weibo has become one of the most mainstream social platforms in China with its weak interactivity and sharing. Users can follow their friends and interact with interested bloggers. When people are interested in an event on the Internet, it will be liked, forwarded, or commented, and spread quickly, resulting in relevant events. At the same time, the same or similar events discussed by everyone form a topic, which has a certain social influence. A hot topic will be formed when a topic is highly concerned or participated by Internet users just like the microblog hot search list. The collective public opinions, emotional attitudes, and values in hot topics form public opinion and have a great impact on public life. Therefore, how to find influential topics from a large number of articles and opinions on microblog is meaningful for the government to grasp the current thoughts and concerns of the people. It is necessary to effectively evaluate the influence of the topic and study the influence of the topic on the society.

The article "ECANP: A Topic Influence Evaluation Model for Hot Topics" was published in 2022. Journal: Comput Intell Neurosci.

However, the openness and inclusiveness of the Internet make it difficult for users to obtain information. Some blogs contain important information, while others contain trivial and meaningless information. People are eager for information that can describe social dynamics. How can we timely obtain the centralized and organized social hot spots and understand the focus information in the vast network? This problem attracts researchers to put forward many effective solutions in the field of topic detection, such as using topic detection method to identify emerging topics in network information flow, and find hot topics through hotness evaluation. Topic hotness evaluation, which can be regarded as a filtering process of hot topics, is used for hot topic discovery, topic recommendation, and topic trend prediction. The hotness of the topic is used to measure the influence of the topic. Traditional influence evaluation methods only consider the frequency of news reports for hotness evaluation. In their opinion, the more news reports contained in one topic, the higher the attention, and the greater the hotness. Or they think that the hotness of the topic is mainly reflected in the number of comments and clicks. Although the influence evaluation method has been improved in some follow-on evaluation algorithms, such as TF-PDF [3–5] hotness evaluation algorithm, which only considers the influence of media on topic attention; literature [6] takes into account the users' attention to topics, but these influencing factors are not comprehensive enough and are not applicable to all fields. Therefore, we are more concerned about how to fully extract the effective information in blog posts and analyze which influencing factors could be quantified as the evaluation factors of hot topics.

The article "ECANP: A Topic Influence Evaluation Model for Hot Topics" was published in 2022. Journal: Comput Intell Neurosci.

Owing to the strong interactivity, fast propagation speed, and easy use of social networks, the network platform will produce a large amount of data every day, forming a lot of topics, which resulting in a rapid update of topic hotness, and the new hot topics will cover the old hot topics. When an event on the website may trigger massive relevant information, forwarding, and comments in a short time, the event will immediately become a hot topic. In addition, because the hotness of the topic varies in different periods of time, and new topics will continue to emerge in the same period of time, especially the topics related to judicial cases and political reports in microblog may last for a long time, but there are not many articles related to the topic produced during this period, so the hotness of the topic will be relatively small. However, if a topic produces extensive relevant articles in a short time, the topic will be more popular. Hot topics have a lifecycle, and they will go through the process from “generation” to “extinction”. Therefore, we can analyze that interactive behavior, topic volume, and time are all significant factors affecting topic hotness.

In order to more accurately evaluate the popularity of topics, this paper proposes an evaluation model of real-time relative influence of topics in social networks (named ECANP), according to the initials of the five indicators---E (Engagement), C (Coverage), A (Activity), N (Novelty), and P (Persistence). Our model will analyze the law of increase and decline of topic hotness from five aspects: user engagement, topic coverage, topic activity, topic novelty, and topic persistence, so as to better distinguish hot topics from cold topics.

The main contributions of this work are summarized as follows.

- We emphasize the relative influence and time attenuation of the topic. At the same time, multiple topics may appear at the same time, and the hotness ranking of topics depends on the relative influence between topics. In addition, topics have a lifecycle. With the passage of time, new topics gradually emerge and old topics are slowly replaced, so the time attenuation characteristics of topics are closely considered in the paper.
- A new model for topic influence evaluation, ECANP, has been proposed, which comprehensively evaluates the relative popularity of topics by integrating user engagement, topic coverage, topic activity, topic novelty, and topic persistence.
- Extensive experiments have been conducted on real datasets to prove the effectiveness of ECANP.

The article "ECANP: A Topic Influence Evaluation Model for Hot Topics" was published in 2022. Journal: Comput Intell Neurosci.

The remainder of this paper is organized as follows.  Section 2 describes the related works.  Section 3 presents the influence evaluation model in detail.  Section 4 constructs experiments to verify the model and analyze the effectiveness of the model. Finally, conclusion is provided in Section 5.

## 2. Related Work

As an important channel of information dissemination and sharing, social networks bear the overload of information. Compared with the early era of lack of information, the biggest difference of social networks is that users can create information while browsing information. Moreover, the online social networking provided by the Internet almost imitates real life. Even if there is no contact between people, the purpose of information communication, sharing and dissemination can be achieved, and this way is more free and flexible. Due to the great participation of users, many subjective blog posts have been formed on the network, and continue to develop into topics, resulting in public opinion, which has a great impact on the public's point of view and life. In order to monitor public opinion in time, find hot topics and extract valuable public opinions from a large number of unorganized and complex data, numerous research scholars devote themselves to the research in this field.

Since 1996, the Defense Advanced Research Projects Agency (DARPA) proposed the concept of Topic Detection and Trace (TDT) for automatically judging the theme of news data flow without human intervention, which has attracted extensive attention, including well-known universities such as IBM Watson Research Center, BBN Company, and Carnegie Mellon University. Companies and research institutions have participated in the evaluation of subsequent TDT. Although domestic research on TDT started relatively late, since National Taiwan University participated in the evaluation of TDT topic detection task in 1999, Peking University, Chinese Academy of Sciences, and Fudan University began to study TDT-related technologies, and put forward many researches using topic detection and tracking to solve the tasks of topic clustering and hot topic discovery, which have achieved prominent results.

The emergence of TDT promotes the discovery and tracking of new events in news reports [7, 8]. The existing topic detection methods mainly focus on the methods based on machine learning [9–13]. For example, literature [14–16] proposes a topic detection method based on incremental clustering to automatically discover and track online news. In reference [17], Ma et al. tracked the online news topics based on the improved vector space model (VSM) model, extracted as characteristics of feature vectors through the lexical chain based on HowNet, and finally used the initial weight and structural weight of the features to construct the semantic vector space model.

The article "ECANP: A Topic Influence Evaluation Model for Hot Topics" was published in 2022. Journal: Comput Intell Neurosci.

Topic detection can undoubtedly help people quickly find out what topics people are discussing from a large number of online articles, but it cannot focus on hot topics, especially when there are many topics and time is limited, it is impossible to choose which part of the more important topics to participate in. Therefore, topic influence assessment is particularly important in hot topic detection tasks.

Hot topic detection is generally divided into two tasks: topic detection and hotness evaluation. Topic discovery depends on topic detection technology, and the generation of hot topics depends on the hotness evaluation method. As for how to measure the hotness of topic, different researchers have successively analyzed the factors affecting the evaluation of topic hotness from different aspects based on the concept of “hot topic”, and all captured the characteristics of topic hotness to varying degrees.

Chen et al. [18] constructed a topic hotness evaluation model based on four factors: media attention, topic competition, topic intensity, and topic cohesion; Deng et al. [19] believed that opinions of comments represented the attitudes of different reviewers towards the topic, and comments with more opinions were hotter. Thus, they not only considered the number of reviews, comments, and publication time, but also took the comment opinion into account to evaluate the hotness of the blog topic; Li et al. [20] divided the factors affecting hotness into internal characteristics and external characteristics. Internal characteristics refer to number of clicks, reply, participating users and topic post, and external characteristics refer to duration time of topic, post source, number of released post, and topic quality. However, these methods do not take into account the characteristics of topic lifecycle.

Zhong [21] sorted out the characteristics of hot topics by analyzing the meaning of topics and hot topics, and proposed a method to extract hot terms that can represent hot topics from text documents based on the two key attributes of hot terms: persistence (the frequency with which a term appears in a set of documents) and topicality (the variation in the frequency of usage of a term over time). Through the distribution and change of hot terms in time, the clustering of hot topics in a given time period can be identified by weighting and applying TF*∗*PDF and aging theory, respectively. Wang et al. [22] extracted the time attribute, report attribute, user attention, and other characteristic parameters of news reports, and established evaluation model of hot topics to evaluate the popularity of clustering topics. Although these methods consider the attenuation characteristics of topic hotness, they do not fully mine the attention of users.

The article "ECANP: A Topic Influence Evaluation Model for Hot Topics" was published in 2022. Journal: Comput Intell Neurosci.

Liu and Hu [22] introduced aging theory while concerned about the inconsistency between media focus and user focus. Assuming that the value of energy attenuation remains unchanged, they use the energy function to express the hotness. However, the lifecycle of different topics is different, and the attenuation degree with time is also different. Therefore, this assumption is unreasonable.

Based on the statistical idea and time characteristics, this paper comprehensively considers the attenuation characteristics of user attention and topics from five aspects, and proposes a new evaluation model of real-time relative influence of topics in social networks by integrating user engagement, topic coverage, topic activity, topic persistence, and topic novelty. The model not only analyzes the user's attention to the topic from the user behavior, but also considers that the influence of the topic is relative. Finally, it also concentrates on the time attenuation characteristics of the topic and considers the topic characteristics in a more fine-grained manner.

## 3. The Proposed Model

In this section, we first introduce the three important concepts involved in this paper. Then, we elaborate on the factors that determine the evaluation model. At last, we propose an influence evaluation model, called ECANP, and present the detailed components of ECANP.

### 3.1. Problem Definition

For ease of understanding, this section gives explanations of important concepts and lists the description of important symbols in Table 1.

**Definition 1 .**

TopicIn Topic Detection and Tracking (TDT) research, a topic is defined as a composition of core events or activity and events or activities directly related to it. An event is something that occurs at a specific time and place, involves some people or things, and may be accompanied by some inevitable results. Specifically, the topic is not a large field (such as the “national two sessions”) or a certain type of event (such as the “Winter Olympics Games”), but a very specific “event”, such as the “Fengxian event”, and then the reports on the “Fengxian event” are considered to be related to the topic of “Fengxian event”. In general, we can simply treat a topic as a collection of several reports related to an event [23].

The article "ECANP: A Topic Influence Evaluation Model for Hot Topics" was published in 2022. Journal: Comput Intell Neurosci.

**Definition 2 .**

Topic HotnessDifferent topics have different effects on the public. When the event forms a topic, some of which will receive more attention and discussion from people for a period of time, while others only get the attention and participation of a few people. According to the different degree of attention and participation received by the topic, it is expressed as the different influence of the topic, which is quantified as the topic hotness. Topic that has a high hotness is called hot topic. Hotness is a relative concept. Ranking according to the hotness of the topic could get the ranking list of hot topics, so as to distinguish hot topics from the rest of the topics.

**Definition 3 .**

Influence EvaluationHow to quantify the impact of a topic is the focus of evaluation. Whether a topic is popular or not depends on the feedback from users. On the basis of the user's feedback on the topic, such as likes, forwards, comments, original microblogs, and other forms of engagement, quantifying the influence generated by the topic as hotness is the influence evaluation.

### 3.2. Key Study

The general process of topic hotness evaluation is shown in Figure 1. The general process consists of four layers: input layer, data layer, model layer, and output layer. The input layer clusters the data required by the model through topic detection and discovery technology, and each topic contains many blog posts belonging to the topic. The data layer is responsible for extracting the evaluation factors of calculation hotness for each topic. The model layer uses the proposed hotness evaluation model to calculate the hotness of each topic. Finally, the hot topic list is generated in the output layer according to the hotness value obtained from the topic.

Targeting the topic influence evaluation problem, we propose a new solution, called ECANP. As shown in Figure 2, the model is divided into five components: i.e., user engagement, topic coverage, topic activity, topic persistence, and topic novelty. We first discuss how the five indicators affect the topic hotness in Section 3.2.1, then present the specific evaluation model, and introduce the calculation details of each component in Section 3.2.2.

#### 3.2.1. Evaluation Factors Analysis of the Topic Hotness

With the development and application of topic detection technology in research and industry, the massive amount of information on the Internet is integrated into orderly and classified modules, which is convenient for users to view other articles related to the topic of an article, that is, they belong to the same topic, so as to form their own opinions. But in reality, we find that even if information is aggregated into topics, the number of topics is still huge and various. If the topics can be sorted according to certain strategies, users will access the information they demand more efficiently and conveniently, thereby meeting the needs of users.

The article "ECANP: A Topic Influence Evaluation Model for Hot Topics" was published in 2022. Journal: Comput Intell Neurosci.

One strategy for ranking topics is to quantify the influence of topics at the topic level, that is, hotness, and rank them according to the hotness of topics. The hotter the topic, the higher the influence, thus the higher the ranking, and vice versa. Different from ordinary topics, hot topics usually have close user attention, wide coverage, high release frequency, and other characteristics. Therefore, we should first determine some factors related to topic hotness, and establish a topic influence evaluation model by analyzing the different effects of various factors on topic influence. As follows, this paper defines five factors related to topic hotness evaluation at the topic level.

*(1) User Engagement*. In online social networks, the formation of hot topics is affected by many factors, but extensive user engagement is the foundation of forming a hot topic. Because only when a certain number of people browse, participate, and pay attention to, the topic will have a certain social influence, thereby attracting more people to be involved. In real life, through face-to-face contact and communication, a large number of people gather and participate in a certain place for a period of time, resulting in an influential activity. The network world is a reflection of the real world. Depending on the dissemination and sharing of the Internet, people can communicate freely across time and space. This is how social networks come into being. Different from the real social interaction, people's participation in online social networking sites is expressed as explicit participation and implicit participation. Publishing original articles, forwarding articles, and liking or commenting on articles are explicit participation behaviors. Browsing and searching related content are the implicit participation behaviors. From the perspective of topic, the explicit feedback and implicit feedback they receive exactly reflect user's attention and participation in the topic. The like behavior shows that the liked content can attract user's attention, cause their resonance, and reflect their favor and appreciation of the content. When users are interested in a blog post, have some opinions, and want to get more information related to content, they tend to give comments, which reflects the user's awareness and interest in the content. When users are approve of the content they are interested in, they will be prompted to forward the content, so that the content can obtain more exposure and share with more people, reflecting users' recognition of the content.

The article "ECANP: A Topic Influence Evaluation Model for Hot Topics" was published in 2022. Journal: Comput Intell Neurosci.

Due to users' explicit feedback is easy to obtain, this paper measures users' engagement through their likes, forwards, and comments on topic articles. The more likes, forwards, and comments, the more attention user pays to the topic, and then topic will be widely spread owing to user's forwarding behavior. Due to user's comment behavior, more users will be appealed to participate in the discussion of the topic, thus expand the dissemination and influence of topic.

*(2) Topic Coverage*. A topic is a collection of seed events and related events. Hot topics usually have a broad user base. They will publish many original articles related to the topic, which makes the number of articles contained in the topic continue to increase. The number of articles contained in a topic reflects the hotness of topic to a certain extent. Compared with the number of articles related to other topics in the same period, the number of articles related to the topic reflects relative influence of the topic. Generally speaking, the topic which has more relevant articles is hotter. The more the number of articles related to a topic accounts for total number of articles on all topics at the same time, indicating that the topic has greater influence than other topics. For instance, if there are 1000 related articles on topic A from its emergence to its demise, but there are 10000 related articles on topic B, we believe that topic A is more popular than topic B in terms of topic coverage.

It can be seen that the number of articles related to topic is an important factor to measure influence of topic. Therefore, the coverage of a specific topic in all topics is of great significance to quantify the hotness of topic.

*(3) Topic Activity*. Articles on social networks (such as microblog) can be regarded as a text stream on the timeline. When a blog post is published, with the attention and participation of users, a certain number of relevant articles will be generated in succession over a period of time to form a topic. If this time period is short, a topic generates a large number of relevant articles, while another topic only generates a small number of articles, the topic with generous relevant articles in a short time will get more attention and higher hotness. Or in another case, if a topic produces many articles, but it is distributed over a long period of time, and the average number to the time unit is small, the hotness value will be smaller than that of the topic that produces many relevant articles in the short term. That is, the more relevant articles on topic are published per unit of time, the more its influence can be reflected. Therefore, as a hot topic, we should not only consider the proportion of the number of articles related to topic, but also take the activity per unit time into account.

The article "ECANP: A Topic Influence Evaluation Model for Hot Topics" was published in 2022. Journal: Comput Intell Neurosci.

Generally speaking, in the whole time period, the more frequently a topic is discussed, the more active the topic is, the more relevant articles it has compared with other topics, and the greater its influence. Therefore, the number of articles produced by the topic per unit time is also one of the major factors affecting topic hotness, thus we can acquire the activity of the topic.

*(4) Topic Novelty*. Hot topics are those topics that are frequently discussed and concerned by the public for a period of time and within a certain range. The hotness of topic will accumulate with the increasing attention of users and media, otherwise it will gradually decay over time, which is consistent with the life cycle of the topic modeled by Liu and Hu [24] based on aging theory. Affected by the “life cycle”, hot topics will go through a process from “generation” to “extinction”. Accordingly, their hotness will change with the change of life cycle and eventually decline naturally. In addition, people prefer new topics and current events to old ones. In particular, with the migration of time, new topics gradually emerge and attract users' new attention, naturally, fewer and fewer people pay attention to the old topics, and the number of articles related to them also decreases. However, more and more attention is paid to the new topics, resulting in the old topics being gradually replaced by the new topics, and gradually fade out of people's memory, and people turn to pay more attention to the development of new topics.

Therefore, the earlier the topic first appears from the current time, the smaller its impact on users and the smaller its hotness value. On the contrary, the closer the topic appears to the current moment, the more active it is, and the more it can draw the attention of users, the higher its contribution to hotness value, and the more likely it is to become a hot topic. Hence, the novelty indicator of topic is obtained by using the attenuation function with number of time unit intervals between current time and first release time of topic.

*(5) Topic Persistence*. Traditional topic hotness evaluation model tends to consider the impact of media attention (i.e., the number of relevant reports) and user attention (i.e., user clicks and participation) on the hotness. Recently, more researchers have considered the characteristics of topic life cycle, but still neglected another property of topic itself, that is topic persistence. A topic always develops with time, and it is not easy for an event to become a topic overnight, which requires magnanimous users' long-term discussion and participation. The longer a topic is discussed and concerned by users, the more it can arouse users' interest, and the more likely it is to attract more users to participate. Nevertheless, some topics are not necessarily discussed every day and have nodal property. Such as the “jiangge incident” that has lasted until now in 2016, which will appear again on the social platform and become a hot topic whenever there is new progress in the case. Consequently, the total number of time units in which topic is continuously discussed in specified time period will be acted as an important indicator to measure topic hotness in this paper.

The article "ECANP: A Topic Influence Evaluation Model for Hot Topics" was published in 2022. Journal: Comput Intell Neurosci.

User engagement is used to calculate the user influence related to topic. Topic coverage is used to calculate the propagation coverage of related topics. Topic activity is used to calculate the activity of related topics. Topic novelty is used to calculate the contribution value of the novelty of related topics to hotness. And topic persistence is used to calculate the time when relevant topics are continuously active on the social platform. Based on the above analysis, the newer the topic, the more public participation and discussion, the wider the coverage, the higher the activity, and the longer the duration, and the more likely topic is to have a high hotness value and become a hot topic. We will propose topic hotness evaluation model in Section 3.2.2, and verify the model through experiments in Section 4.

#### 3.2.2. Topic Hotness Evaluation Model: ECANP

Based on the factors related to topic influence evaluation analyzed in the previous section, it can be concluded that user engagement, topic coverage, topic activity, topic persistence, and topic novelty can be used as evaluation factors to quantify a topic influence. Following the above indicators, multiple topics will be generated successively in a period of time, and the relative influence of each topic is quantified as the hotness evaluation. Because topic coverage, topic activity and topic persistence belong to topic attributes, besides, topic attributes, and user participation will gradually weaken with the passage of time, so the operation of influence evaluation integrating five indicators can be formulated as follows:

(1) $$\begin{array}{c} {\text{Hot}}_{j}=\left(\begin{array}{c} \text{Engagement}\left(j\right)+\text{Coverage}\left(j\right)*\text{Activity}\left(j\right)\\ {}*\text{Persistence}\left(j\right) \end{array}\right)*\text{Novelty}\left(j\right), \end{array}$$

where Engagement (*j*) denotes the user engagement in topic *j*. We first employ the entropy weight method to determine the weight of each indicator affecting user participation, and then apply the sum aggregator to aggregate the impact of the three indicators for expressing the influence of users' participation behavior on the topic. Utilizing entropy weight method to determine the indicator weight can be divided into two steps: data standardization processing and entropy weight determination of the indicator.

*(1) Data Standardization Processing*. We consider that there are *m* topics in a period of time, and the user engagement factor of each topic has *n* measurement indicators. Let *R* ∈ *R*^*m*×*n*^ denote the judgment matrix, and build *R* before standardizing the data:

(2) $$\begin{array}{c} R={\left(r_{ji}\right)}_{m\times n},\;\left(j=1,2,\ldots ,m;i=1,2,\ldots ,n\right). \end{array}$$

Then, for the sake of eliminating the adverse effects caused by singular sample data, we employ maximum and minimum normalization to standardize the judgment matrix *R* to acquire the standard data limited in the range of [0, 1]:

(3) $$\begin{array}{c} b_{ji}=\frac{r_{ji}-r_{\min}}{r_{\max}-r_{\min}}, \end{array}$$

where

(4) $$\begin{array}{c} r_{\min}=\min\left(r_{1i},i,\ldots ,r_{mi}\right), \end{array}$$

(5) $$\begin{array}{c} r_{\max}=\max\left(r_{1j},r_{2j},\ldots ,r_{mj}\right). \end{array}$$

In equation (2), *m* represents the number of topics, *n* denotes the number of indicators to measure user engagement, and *r*_*ji*_ means value of the *i*-th indicator of the *j*-th topic;

In equation (3), *r*_max_ and *r*_min_ represent the maximum and minimum values of the number of likes, forwards, and comments of the relevant articles on different topics under the same measurement indicator, respectively. And *b*_*ji*_ stands for maximum and minimum normalization value of *r*_*ji*_.

*(2) Entropy Weight Determination of the Indicator*. We define the weight of all likes, forwards, and comments of each topic as follows:

(6) $$\begin{array}{c} W={\left(w_{i}\right)}_{1\times n}, \end{array}$$

where

(7) $$\begin{array}{c} w_{i}=\frac{1-H_{i}}{n-\sum_{i=1}^{n}H_{i}}. \end{array}$$

According to the definition of entropy, the weight of all measurement indicators can be determined:

(8) $$\begin{array}{c} H_{i}=-\frac{1}{\ln\;m}\sum_{j=1}^{m}f_{ji}\ln\;f_{ji},\;\left(0<H_{i}<1\right), \end{array}$$

(9) $$\begin{array}{c} f_{ji}=\frac{1+b_{ji}}{\sum_{j=1}^{m}\left(1+b_{ji}\right)}\;,\;\left(j=1,2,\ldots ,m;i=1,2,\ldots ,n\right), \end{array}$$

where *f*_*ji*_ denotes the proportion of the *j*-th indicator in the *i*-th topic.

The article "ECANP: A Topic Influence Evaluation Model for Hot Topics" was published in 2022. Journal: Comput Intell Neurosci.

Through analysis, we can know that if the value of *f*_*ji*_ in equation (8) is 0, ln 0 will inevitably occur. For solving this problem, our paper adopts the following formula amend *f*_*ji*_′.

(10) $$\begin{array}{c} f_{ji}^{\prime }=\frac{b_{ji}}{\sum_{j=1}^{m}\left(b_{ji}\right)},\;\left(j=1,2,\ldots ,m;i=1,2,\ldots ,n\right). \end{array}$$

In line with above contents, the weight of each measurement indicator under each topic can be calculated. Then, the final user engagement can be obtained through the sum aggregator.

Based on the analysis of topic influence factors in Section 3.2.1, we finally determine that user engagement is affected by three indicators: likes, forwards, and comments. Therefore, this paper calculates the weight of these three indicators and aggregates them through equation (11):

(11) $$\begin{array}{c} \text{Engagement}\left(j\right)=\alpha \times L_{j}+\beta \times R_{j}+\gamma \times C_{j}. \end{array}$$

Then, coverage (*j*) denotes the topic coverage in topic *j*, which is calculated based on the proportion of the number of articles related to topic *j* in all topic articles, that is,

(12) $$\begin{array}{c} \mathrm{Coverage}\left(j\right)=\exp\frac{Q_{j}}{Q}. \end{array}$$

Next, activity (*j*) denotes the topic activity in topic *j*. By calculating the number of articles on topic *j* in unit time, we can obtain the activity of the topic *j*, that is,

(13) $$\begin{array}{c} \mathrm{Activity}\left(j\right)=\ln\frac{Q_{j}}{T_{j}}. \end{array}$$

Similarly, novelty (*j*) denotes the topic novelty in topic *j*. According to the difference of time units between current time and the time when the topic *j* was first published, the novelty indicator of topic *j* is obtained:

(14) $$\begin{array}{c} \mathrm{Novelty}\left(j\right)={\left(\nabla t\left(j\right)+1\right)}^{-k}, \end{array}$$

(15) $$\begin{array}{c} \nabla t\left(j\right)=t_{t}-t_{p}, \end{array}$$

where *t*_*t*_ is current time (for example, if the collected experimental data is from April 1 to April 30, 2020, the current time is April 30), *t*_*p*_ is the first release time of topic *j*, and ∇*t*(*j*) is the difference of time units between the current time and the first release time of the topic, time in days. *k* is the attenuation factor, which controls the attenuation rate of topic *j* over time. The larger ∇*t*(*j*), the smaller novelty (*j*), and the less contribution of this indicator to hotness.

Finally, persistence (*j*) denotes the topic persistence in topic *j*. According to the duration of the topic *j* in the life cycle and the proportion of the number of units in the whole topic monitoring time, the persistence of the topic is obtained:

(16) $$\begin{array}{c} \mathrm{Persistence}\left(j\right)=\frac{n_{u}}{n}, \end{array}$$

the total duration *n*_*u*_ of topic *j* is obtained by equation (17), that is,

(17) $$\begin{array}{c} n_{u}=n_{e}-n_{b}, \end{array}$$

where *n*_*u*_ is the number of time units in which topic *j* is reported and discussed, time in days. *n*_*e*_ indicates when the topic dies, and *n*_*b*_ represents when the topic arises.

The article "ECANP: A Topic Influence Evaluation Model for Hot Topics" was published in 2022. Journal: Comput Intell Neurosci.

Further, the influence evaluation of topic *j* in equation (1) can be obtained by aggregating the above five indicators. Therefore, the hotness value Hot_*j*_ of topic *j* is described as follows:

(18) $$\begin{array}{c} {\text{Hot}}_{j}=\left(\left(\alpha \times L_{j}+\beta \times R_{j}+\gamma \times C_{j}\right)+\exp\frac{Q_{j}}{Q}\times \;\ln\frac{Q_{j}}{T_{j}}\times \frac{n_{u}}{n}\right)\times {\left(\nabla t\left(j\right)+1\right)}^{-k}, \end{array}$$

where *k* is the attenuation coefficient.

#### 3.2.3. Interpretability Discussion of the Model

Entropy weight method is an objective method to determine the weight, which has certain accuracy compared with subjective methods such as analytic hierarchy process. Moreover, the weight value determined by this method could be modified, which determines its high adaptability. The formula for calculating entropy value in entropy weight method was put forward by information scientist Shannon. When the data is more dispersed and the entropy is smaller, it can be considered that the data contains more information, so the weight is larger. According to Section 3.2.1, a topic will get users' likes, forwards, and comments. These behaviors represent users' different degrees of preference for the topic and reflect users' engagement. Therefore, in order to identify the contribution of user behavior factors to users' engagement, entropy weight method is used to calculate their weight. After that, user engagement can be obtained by weighted summation of behavior factors.

In addition to considering users, the attributes of the topic itself, including text attributes and time attributes, should not be ignored. The text attributes of topic include topic coverage and topic activity, and the time attributes comprise topic novelty and topic persistence. In a series of blog posts, the more blog posts related to the topic, the wider their coverage, which is expressed as the proportion of the number of blog posts related to the topic in the total blog posts, i.e., *Q*_*j*_/*Q*. Over a period of time, the more blog posts related to the topic, the higher their frequency, and the easier it is to catch the user's eye, which is expressed as the number of blog posts related to the topic in unit time, i.e., *Q*_*j*_/*T*_*j*_. Generally, (*Q*_*j*_/*Q*) ∈ (0,1].

The article "ECANP: A Topic Influence Evaluation Model for Hot Topics" was published in 2022. Journal: Comput Intell Neurosci.

The topic of sustainability that people pay attention to can gain higher hotness. The longer the topic lasts, it means that people are more interested in the topic; the topic continues to ferment and has a greater impact on more users. We use the proportion of the number of time units in which the topic is reported to the total time units to express topic persistence, i.e., *n*_*u*_/*n*.

Topics are always updated iteratively. “From emergence to extinction” is a process that every topic will experience. Over time, the contribution of each attribute of the topic to its hotness is gradually weakening, as described by the aging theory [22]. The attenuation degree of topic determines the novelty of topic, which depends on two factors, including the time span of topic and the attenuation factor. For the attenuation function, we choose the inverse proportional function of time factor, because its value range is larger, the attenuation degree of new topic and old topic is clearly distinguished, and the attenuation is stable.

## 4. Experiments and Analysis

We testify our proposed model by conducting extensive experiments on real-world corpus, aiming to answer the following key questions.

- Q1: How can the topic influence evaluation model effectively explain the topic hotness?
- Q2: How does ECANP perform compared with state-of-the-art influence evaluation models?
- Q3: Can five indicators (i.e., user engagement, topic coverage, topic activity, topic persistence, and topic novelty) reasonably explain the impact on ECANP?

### 4.1. Datasets

To demonstrate the performance of our method ECANP and compare it with the baseline methods, a corpus of microblog articles is adopted. Six topic data are used for experiments to verify the universal applicability of the model ECANP in this paper. The topic names are shown in Table 2. The data in the datasets comes from the judicial cases provided by Yifang, and the time range of topic is from December 14, 2020 to January 11, 2021, with an overall data volume of more than 50000 pieces. This paper evaluates the influence of topic by utilizing the six topics that users have participated in for a long time provided by Yifang and the analysis of the hotness of each topic. Before using the data, we check the dataset through conventional data preprocessing method to remove the unusable or invalid data. The specific data statistics are shown in Table 3.

### 4.2. Experimental Settings

#### 4.2.1. Evaluation Metrics

Since there is no unified evaluation indicator for topic influence evaluation, in order to prove the effectiveness of the model, this paper consulted a large number of relevant literature. Inspired by [19], we finally determined to carry out experimental verification from three aspects, namely the effectiveness of model (Effectiveness verification, abbreviated as EFVC), the comparison of ability to distinguish hot and cold topics with the baseline evaluation methods (Ability to distinguish hot and cold topics, abbreviated as ADHCT), and the impact of each evaluation indicator on the model (Control variable analysis, abbreviated as CVA), corresponding to the above three questions.

The article "ECANP: A Topic Influence Evaluation Model for Hot Topics" was published in 2022. Journal: Comput Intell Neurosci.

#### 4.2.2. Baselines

To support the effectiveness of ECANP model, we compare it with the following five baseline models, in which the first four models are verified with the same and only one dataset, and the fifth is verified with the six datasets used in this paper due to the particularity of its method. In addition, some comparison models do not have a name, for ease of display, we give a name according to the naming method in this paper. The experimental settings of proposed model and baselines are introduced in the next subsection.

- BHEM-TOA [20]: This is a blog hotness evaluation model based on comment opinion analysis, which realize blog hotness evaluation through the number of reviews, comments, publication time, and the opinioned comments.
- FSTCC [1]: Such a model is proposed to calculate the hotness value of online news topics about the emergency events, which considers reporting frequency of topics, the number of report sources, time property, click rates of users, and the number of comments.
- HFTC [24]: This is a method to evaluate topic hotness by exploiting the frequency of topic tags. Specifically, it takes several keywords with the highest probability of occurrence in topic as the tag set, calculates topic hotness by using topic tag frequency without relying on any information other than the text itself, and finally determines the latent topic with the highest hotness value as hot topic in the unified network.
- IEFE [21]: This is a topic hotness evaluation model, where considers the internal and external factors impacting the hotness. The characteristics of hot topics are analyzed by internal factors such as number of clicks, comments, and user participation, as well as external factors such as topic duration, topic quality, and topic concentration.
- DMCBF [19]: This model is based on decay, media attention, topic competition, and topic cohesion. The hotness value of each day is calculated through the energy function, and the accumulation of hotness value of each day is regarded as the accumulated hotness of the topic after *d* days.

The article "ECANP: A Topic Influence Evaluation Model for Hot Topics" was published in 2022. Journal: Comput Intell Neurosci.

#### 4.2.3. Experimental Settings

For the three experiments in the next section, we adopt different settings and data processing methods.

For the first experiment, we implemented our ECANP model in six experimental datasets, presenting the hotness results of each topic, and the results of some influencing factors.

For the second experiment, the settings of comparison models are divided into two categories. To realize the comparison between our proposed method and the first four models, we selected Topic 1 in datasets for experiment. Firstly, we clustered multiple subtopics and topic names under Topic 1 through topic detection method and topic name detection, and then ran ECANP and four baseline models respectively to calculate the hotness of each detected subtopic. For comparability, the hotness of all models is normalized in the range of 0–100. The normalization formula is equation (19). Due to the particularity of the fifth comparison model, we regard each dataset as a separate topic, divide each topic according to the number of days, and get the relevant articles of the topics in each day. ECANP and DMCBF are used to calculate the hotness of six topics respectively. Finally, we select the hotness value of the five hottest topics and the five coldest topics obtained by the first four models, as well as the hotness value of all topics of the last model, contrast ECANP model with them respectively, and compare the performance according to the judgment formula of hot and cold topic discrimination ability:

(19) $$\begin{array}{c} {\text{Hot}}_{j}\_\text{norm}=\frac{\ln\;{\text{Hot}}_{j}}{\ln\;\max\;\left({\text{Hot}}_{1},{\text{Hot}}_{2},\ldots ,{\text{Hot}}_{j}\right)}. \end{array}$$

For the third experiment, to clearly see the change of topic hotness and its indicators over time, we divided the life cycle of topic into 8 time periods, obtained the articles related to the topic in each time period, and took the last time point of the time period as the coordinate label.

The settings of each baseline model are as follows.

  BHEM-TOA: we removed the part of text comments in this baseline method, because the author evaluates the hotness of Blog websites, which is composed of the hotness of multiple topics. Multiple topics under a website do not distinguish comments, so it is set as a constant in this paper, and its value is 0.
  FSTCC: different hotness evaluation methods use different indicators for different scenarios. Owing to there is no report sources in our datasets used in this baseline method, such information is ignored. In addition, the time interval used by the author is the difference between the current time and the topic publishing time, but the experimental results show that the publishing time of the topic in the dataset is too long from the current time, and the time attenuation is quite large, resulting in the hotness value of 0. Therefore, this paper uses the duration of the topic instead of the current time in the paper. The time interval is set to 1 day.
  HFTC: the author applies the proposed model to cross social networks. To compare with our method, only the single platform topic hotness evaluation in author's paper is used.
  IEFE: in the implementation of this method, since there are no number of clicks in our datasets, this item and the publishing sources are ignored, and the number of microblog articles is used to replace the number of user participation.
  DMCBF: the time used in the model is in days.

The article "ECANP: A Topic Influence Evaluation Model for Hot Topics" was published in 2022. Journal: Comput Intell Neurosci.

In equation (18), the attenuation coefficient is set to 0.1.

### 4.3. Experimental Results and Analysis

#### 4.3.1. Result 1: Validity Verification (Answer the Mentioned Q1)

Based on the statistical experimental data in Section 4.1, we use the topic hotness evaluation model proposed in this paper to evaluate the hotness of all topics in the dataset, calculate the hotness value of each topic, and rank them according to their hotness value. As shown in Table 4, it presents the model results and topic ranking.

Due to the long real name of the topic, for convenient representation and viewing, the topic name is listed in the form of “topic + number” in the charts in this paper. The actual correspondence between topic name mark and real topic name is shown in Table 2.

In Table 4, the left part shows the hotness value of each topic and its corresponding ranking results, and the right part lists the topic ranking results from high to low according to the hotness value. From the above results, we can conclude that among the six groups of experimental data, Topic 4 has the highest hotness, while Topic 2 has the lowest hotness. Since the hotness of topic is relative over a period of time, the influence of topic with the highest hotness is quantified as 100. By sorting the relative influence of topics, the topic ranking table is obtained.

In this part of the experiment, to validate the effectiveness of our topic influence evaluation model, we evaluated and analyzed the hotness values of six topics. ECANP first extracts the number of forwards, comments, related blog posts, topic duration, hotness evaluation time period, and current time of each topic, then utilizes these information to calculate the hotness of each topic through each indicator calculation method and hotness evaluation formula proposed in Section 3.2.2, and finally presents the histogram of the number of forwards, comments, and blog posts of each topic in Figure 3; meanwhile, the hotness value of each topic is also shown in Figure 3 as a line chart. It can be seen that the change trend of topic hotness value is consistent with the trend of forwards, comments, and blog posts. For example, on the whole, the number of forwards, comments, and blog posts of Topic 2 is less than that of Topic 1, accordingly, the hotness value of Topic 2 is also less than that of Topic 1, and so on; from the perspective of single factor, the change trend of forwarding number from Topic 1 to Topic 6 is “down-up-up-down-down”, correspondingly, the change trend of topic hotness is the same, and other single factor analysis of topics is followed by analogy. In particular, the number of comments of Topic 4 is greater than that of Topic 1, but the hotness value of Topic 4 is less than that of Topic 1, which is due to Topic 1 is more novel than Topic 4. Combined with entropy weight method and hotness evaluation formula, it is concluded that the hotness value of Topic 1 is slightly higher than that of Topic 4.

The article "ECANP: A Topic Influence Evaluation Model for Hot Topics" was published in 2022. Journal: Comput Intell Neurosci.

The ranking of hot topics given by ECANP model is the same as expected, which shows that the topic hotness evaluation model proposed by this paper is reasonable and effective.

#### 4.3.2. Result 2: Performance Comparison (Answer the Mentioned Q2)

In this section, we contrast the performance of our ECANP with five baselines, compare their ability to distinguish hot topics from cold topics. Note that, for the baseline BHEM-TOAm FSTCC, HFTC and IEFE, we conduct experiments on the same topic, regard a topic as an event, use the clustering algorithm to obtain the subtopics under topic, and calculate and distinguish the hotness of subtopic. The experimental flow is shown in Figure 4, and then reports the performance of these baselines on the topic. For the DMCBF model, we use the six topics used in this paper to verify, then calculate the hotness of each topic, and report their performance.

Tables 5–8 indicate the experimental results of our method and five baselines, respectively. The table shows the results using equation (20) to normalize, where in Tables 5 and 6, *α* of the ECANP, FSTCC, and HFTC model is set to 0.001, the BHEM-TOA model is set to 0.1, and the IEFE model is set to 0.0001. In Tables 7 and 8, *α* of the ECANP is 0.00001, and *α* of the DMCBF is 1. As shown in Tables 5, 6, and 8, for the topic hotness evaluated by different methods, we use equation (21) to calculate the hotness distance [25] between topics.

Table 9 shows the subtopic names generated in the comparative experiment between ECANP and BHEM-TOA, FSTCC, HFTC, and IEFE. It can be seen from the results that the performance of our method in distinguishing hot topics from cold topics is better than the baselines, exceeding the performance of the optimal baseline model by 0.008%. This is because we make good use of indicators of five dimensions and effectively combine user characteristics and topic attributes. The results show that our method can better identify hot topics and cold topics, making hot topics more popular and cold topics less popular.

(20) $$\begin{array}{c} \text{norm}\_{\text{Hot}}_{j}=\frac{e^{{\text{Hot}}_{j}\times \alpha }-e^{-\left[{\text{Hot}}_{j}\times \alpha \right]}}{e^{{\text{Hot}}_{j}\times \alpha }+e^{-\left[{\text{Hot}}_{j}\times \alpha \right]}}, \end{array}$$

(21) $$\begin{array}{c} \text{Dist}\left(\text{HT},\text{CT}\right)=\frac{\sum_{i=1}^{5}{\left(H^{ht\left(i\right)}-H^{ct\left(i\right)}\right)}^{2}}{\sum_{i=1}^{5}{\left(H^{ht\left(i\right)}\right)}^{2}+\sum_{i=1}^{5}{\left(H^{ct\left(i\right)}\right)}^{2}}, \end{array}$$

where *H*^*ht*^ is the hotness of hot topic *ht* and *H*^*ct*^ is the hotness of cold topic *ct*.

The article "ECANP: A Topic Influence Evaluation Model for Hot Topics" was published in 2022. Journal: Comput Intell Neurosci.

#### 4.3.3. Result 3: Case Study of ECANP (Answer Q3)

Obviously, the user attention and topic attributes in different time periods are not invariable, which enable the hotness of each topic varying with time. In order to clearly show that the change of topic hotness over time is affected by relevant influencing indicators, Figure 5 displays each relevant indicator value and topic hotness of each topic in different time periods of its life cycle. The figure (a–f) reflects the change trend of each indicator and hotness value of six topics in the form of broken line diagram, respectively. Note that the life cycle of each topic is different, and some have long life cycles and some have short life cycles. If the results are displayed at a unified time interval, the graph will be very unsightly and affect the intuition. Therefore, in order to facilitate viewing the results, each topic adopts the same number of time nodes, that is, the time interval of each topic is different, which does not affect the experimental results.

As shown in Figure 5, for each topic, the values of each indicator and topic hotness change in each period. Taking (c) in Figure 5 as an example, the hotness value of Topic 3 at the first time point is 0, while the hotness value rises in the next time period, which means that the topic is still in the embryonic stage at the first time point, and then it obtains extensive user attention and participation, and reaches the hottest at the second time point. With the passage of time, the user attention and the value of topic attributes decrease, resulting in the decrease of topic hotness. At the sixth time node, the trend of user engagement, topic persistence, topic coverage, and topic activity have increased, and the trend of topic hotness is also rising. This shows that proactive user participation, lasting and active topic discussion, and extensive topic coverage will bring about high hotness of a topic and produce great influence. Although the novelty (purple line) and persistence (red line) of Topic 3 gradually increase as time goes on, the change range is very small, so it has little impact on the hotness of the topic. (Note, in the figure, since the values of these two indicators are close, the two lines almost coincide.) On the contrary, if the topic novelty and topic persistence change greatly in different time periods, it will have a great impact on the topic.

The article "ECANP: A Topic Influence Evaluation Model for Hot Topics" was published in 2022. Journal: Comput Intell Neurosci.

The hotness value of topic is jointly determined by various factors such as the forwarding, comments, and publishing time of the topic-related articles, including user characteristics and topic attributes. Due to the large base of users' forwarding, comments, and other behaviors, and the topic is generated almost at the same time period, the user engagement has a great impact on the final hotness of the topic.

ECANP relatively comprehensively analyzes the influencing factors of topic hotness, and makes full use of the factors such as the number of comments, the number of forwarding, the number of articles, and the release time to evaluate the topic hotness from five indicators. This method can effectively quantify the influence of topics and reflect the impact of user participation, topic coverage, topic activity, topic persistence, and topic novelty on the hotness evaluation results. It is more reasonable and practical for guiding topic ranking.

## 5. Conclusion

In this paper, we analyzed the relative influence and time attenuation characteristics of topics and hot topics, as well as each indicator affecting the topic hotness according to the reality that the influence of a topic is relative, not absolute. The topic hotness is measured from five indicators: user engagement, topic coverage, topic activity, topic persistence, and topic novelty, which involves the number of comments, number of microblog articles, and time attenuation characteristics of blogs in the topic, and establishes a topic hotness evaluation model that could quickly aggregate hot topics and evaluate the influence of hot topic. In the experimental stage, we propose to verify the topic hotness evaluation performance from three aspects. Through effectiveness analysis, baseline method performance comparison, and indicator impact analysis, we realize the effective verification and analysis of the topic influence evaluation method proposed in this paper. The results show that ECANP model can effectively evaluate the influence of topics in a period of time, and give a reasonable topic ranking according to its hotness value. Our model involves the calculation of five indicators, but experiments show that the model is low complexity, time-consuming, and easy to understand. The computational complexity will not increase exponentially with the increase of the number of blogs, but linearly with the increase of topics.

The article "ECANP: A Topic Influence Evaluation Model for Hot Topics" was published in 2022. Journal: Comput Intell Neurosci.

Nevertheless, the results of this study have to be seen in light of some limitations. The first is that the research results of this paper calculate the relative influence of topics. Since this paper proposes that it is more meaningful to study whether one topic is more hot than another topic for topic hotness ranking, we are studying the relative influence of topics, which requires the participation of multiple topics, considering the impact of different topics, and finally giving the topic popularity ranking, rather than just calculating the absolute influence of a specified topic. The second limitation relates to the evaluation method of topic influence specifically designed for single domain and single platform in this paper, which has not yet involved cross-domain social platforms.

In view of the above limitations, we will solve them in future work. On the one hand, we will continue to explore the nature of topic and the characteristics of network public opinion. Through the analysis of the multidimensional characteristic attributes of topic, we will find more valuable information. Combined with the high-quality topic propagation influence structure, we will design a more effective topic hotness evaluation model, test the evaluation performance of different topic characteristic models, and realize the evaluation method using the law of topic propagation influence. On the other hand, because of its heterogeneity, multisource and high capacity, cross-domain social platforms have aroused widespread interest and posed many challenges, we will further study the use of multiplatform information features to beyond the evaluation of single platform topic influence.

## Figures and Tables

**Figure 1:** The general process of topic hotness evaluation.

**Figure 2:** The overall framework of ECANP for topic hotness evaluation.

**Figure 3:** Comparison of the number of some indicators and hotness value of different topics.

**Figure 4:** Data processing flow in comparison test.

**Figure 5:** The trend chart of topic indicators and hotness over time.

The article "ECANP: A Topic Influence Evaluation Model for Hot Topics" was published in 2022. Journal: Comput Intell Neurosci.

**Table 1:** Symbols and description used in this paper.

Symbols	Description
*α*	Weight of likes to user engagement
*β*	Weight of forwarding number to user engagement
*γ*	Weight of comment numbers to user engagement
*L*_*j*_	Total likes of topic *j*
*R*_*j*_	Total forwards number of topic *j*
*C*_*j*_	Total comment number of topic *j*
*Q*_*j*_	The number of articles related to topic *j*
*Q*	Total number of articles on all topics
*T*_*j*_	Duration, that is, the time from the appearance to the end of the topic *j*
*n*_*u*_	The number of time units in which the topic was reported like day or month
*n*	The number of time units segmented from the earliest release time of all topics to the acquisition time
∇*t*(*j*)	The number of time units between the current influence evaluation time and the topic release time

**Table 2:** The correspondence between topic name mark and real topic name.

Topic name mark	Real topic name
Topic 1	The murderer of the passion fruit girl case was commuted to death
Topic 2	Murder with a knife in Kaiyuan, Liaoning
Topic 3	Peking University Wu Xieyu's mother killing case opens
Topic 4	The case of Lao Rongzhi in Nanchang, Jiangxi Province was opened
Topic 5	Henan “9-year-old Lao Lai case”
Topic 6	Lai Xiaomin was sentenced to death in the first instance

**Table 3:** Statistics of the datasets.

Topic	Forwards	Comments	Blogs	Start time	End time	Duration (days)
Topic 1	55707	43621	8288	2020/12/28 0 : 00	2020/12/31 23 : 59	4
Topic 2	6785	11576	3520	2020/12/27 0 : 00	2020/12/31 23 : 59	5
Topic 3	16311	32170	6088	2020/12/23 0 : 00	2020/12/30 23 : 59	8
Topic 4	26780	70562	15371	2020/12/21 0 : 00	2020/12/30 23 : 59	10
Topic 5	17966	31265	11894	2020/12/14 0 : 00	2020/12/20 23 : 59	7
Topic 6	15971	20406	6578	2021/1/5 0 : 00	2021/1/10 23 : 59	6

**Table 4:** Results of algorithm model.

Topic name	Hotness value	Ranking	Top	Ranking list of hot topic	Hotness value
Topic 1	100	1	Top 1	Topic 1	100
Topic 2	83.35	6	Top 2	Topic 4	99.64
Topic 3	92.85	4	Top 3	Topic 5	92.99
Topic 4	99.64	2	Top 4	Topic 3	92.85
Topic 5	92.99	3	Top 5	Topic 6	90.11
Topic 6	90.11	5	Top 6	Topic 2	83.35

**Table 5:** Performance comparison of our model and baselines (part one).

Topic label	Topic description	ECANP (ours)	Topic description	BHEM-TOA
		Hotness		Hotness
HT1	①	100.0	①	26.4781
HT2	②	99.9504	②	6.1957
HT3	④	86.5919	③	3.1946
HT4	③	77.0561	④	1.9596
HT5	⑤	29.0486	⑤	1.1666
CT1	⑨	0.0004	⑨	0.0009
CT2	⑩	0.0004	⑩	0.0009
CT3	⑪	0.0004	⑪	0.0009
CT4	⑫	0.0004	⑫	0.0009
CT5	⑬	0.0004	⑬	0.0009

Dist (HT, CT)		0.9999908339562471		0.9999070183251324

**Table 6:** Performance comparison of our model and baselines (part two).

Topic label	Topic description	FSTCC	Topic description	HFTC	Topic description	IEFE
		Hotness		Hotness		Hotness
HT1	①	28.694	①	99.8995	①	99.9984
HT2	③	25.8758	②	15.355	②	97.0389
HT3	②	13.0456	③	15.0499	④	57.737
HT4	⑧	3.7081	⑦	7.8471	③	51.934
HT5	⑲	3.4714	⑳	7.2633	⑤	18.9157
CT1	⑭	0.0905	⑨	0.1	⑫	0.021
CT2	⑩	0.0905	⑭	0.1	⑮	0.021
CT3	⑪	0.0905	⑩	0.1	⑯	0.021
CT4	⑬	0.0905	⑪	0.1	⑰	0.021
CT5	⑫	0.0905	⑬	0.1	⑱	0.021

Dist (HT, CT)		0.991984356		0.99724503648		0.99947001200

The article "ECANP: A Topic Influence Evaluation Model for Hot Topics" was published in 2022. Journal: Comput Intell Neurosci.

**Table 7:** The result of our model and DMCBF.

Topic name	ECANP	DMCBF
Topic 1	19.338433668350692	88.19006162822104
Topic 2	3.582932515952112	27.3980491541227
Topic 3	9.41422561422112	79.2579948124188
Topic 4	18.66498030322313	74.4511671473541
Topic 5	9.554358308112763	99.90728389941798
Topic 6	7.128933737362833	31.796818192414495

**Table 8:** Performance comparison of our model and baselines.

	ECANP		DMCBF	
	Ranking	Hotness	Ranking	Hotness
HT1	Topic 1	19.338433668350692	Topic 5	99.90728389941798
HT2	Topic 4	18.66498030322313	Topic 1	88.19006162822104
HT3	Topic 5	9.554358308112763	Topic 3	79.2579948124188
CT1	Topic 3	9.41422561422112	Topic 4	74.4511671473541
CT2	Topic 6	7.128933737362833	Topic 6	31.796818192414495
CT3	Topic 2	3.582932515952112	Topic 2	27.3980491541227
	Dist (HT, CT)	0.276654078917006	Dist (HT, CT)	0.2079302077825828

**Table 9:** The correspondence between topic label and real subtopic name.

Subtopic name	Topic label
The murderer of the passion fruit girl case was commuted to death	①
Yang Guangyi, the defendant in the passion fruit girl case, was sentenced to death	②
Passion fruit girl's mother responded to the murderer's death sentence	③
Niu Bo, Chaohua	④
Sulfuric acid boy	⑤
Record the process of China's rule of law society bit by bit	⑥
Short comment on court newspaper	⑦
‘LOEWE'	⑧
Xiao He said something	⑨
Yan Mu 1	⑩
Yan Mu 2	⑪
Nothing 1	⑫
Yan Mu 3	⑬
What can you do	⑭
Nothing 2	⑮
Nothing 3	⑯
Nothing 4	⑰
Nothing 5	⑱
Guangxi Yang Guangyi's rape case was retried and sentenced to death	⑲
Nanjing Denghuang 728 extravagant lighting show	⑳

## Data Availability

The data used to support the findings of this study are available from the corresponding author upon request.
